The article "SPOCK2 Promotes the Malignant Behavior of Ovarian Cancer via Regulation of the Wnt/β-Catenin Signaling Pathway" was retracted in 2024. Reasons: signs of a paper mill; suspected computer-generated content; unreliable results or conclusions; concerns about the data.

# SPOCK2 Promotes the Malignant Behavior of Ovarian Cancer via Regulation of the Wnt/*β*-Catenin Signaling Pathway

**DOI:** 10.1155/2022/9223954

**Published:** 2022-09-23

**Authors:** Shanshan Zhao, Haiyan Liu, Mingying Fan

**Affiliations:** ^1^Obstetrical Department, Taian City Central Hospital, Taian, China; ^2^Ultrasonic Diagnosis and Treatment Center, Taian City Central Hospital, Taian, China; ^3^Gynecology Department, The Second Affiliated Hospital of Shandong First Medical University, Taian, China

## Abstract

**Background:**

Ovarian cancer (OC) is a common clinical gynecological disease, which seriously threatens women's health and life. We investigated the roles of SPOCK2 in OC and its associated molecular mechanism in the current study.

**Methods:**

The expressions and prognostic value of SPOCK2 in OC were identified using the clinical data and data from the GEPIA database. Then, SPOCK2 silence was implemented to search functions of SPOCK2 in OC cells. CCK-8 was used to examine cell proliferation. Cell apoptosis was detected by flow cytometry. The OC cell invasion and migration were evaluated by transwell assays.

**Results:**

Overexpressed SPOCK2 was identified in OC, which was correlated with poor prognosis and a shorter survival rate. SPOCK2 downregulation significantly suppressed OC cell proliferation, migration, and invasion, and cell apoptosis was markedly promoted by SPOCK2 silence. Meanwhile, SPOCK2 knockdown could effectively suppress Wnt/*β*-catenin.

**Conclusion:**

SPOCK2 exerted crucial functions in OC progression and could serve as a promising candidate for OC targeted therapy.

## 1. Introduction

Ovarian cancer (OC) is one of the common malignancies of the female reproductive system [1]. A recent study showed that ovarian cancer accounts for 3.4% of the 9.2 million new cancer cases in women worldwide in 2020, as well as 4.4 million female cancer deaths, of which ovarian cancer accounts for 4.7% [2]. OC is the eighth leading cause of malignancy incidence and death in women [3]. Most OC patients are at advanced stages when detected due to the insidious onset of OC and the lack of early diagnosis and effective screening methods, so the prognosis is still poor [4]. Currently, the treatment of ovarian cancer is mainly based on surgery combined with chemotherapy, and most ovarian cancer patients are sensitive to platinum-based chemotherapy, but some patients still have recurrence after complete remission with first-line treatment [5]. Moreover, with the increase in chemotherapy cycles, the time interval of recurrence gradually shortens, and the dose-limiting toxicity of chemotherapeutic drugs increases, eventually leading to the decrease in patients' sensitivity to drugs, leading to treatment failure and death of ovarian cancer patients [6]. This is the main reason for treatment failures and deaths of OC patients. The development of drug resistance is an important cause of recurrence and death, but there is no effective treatment for platinum-resistant patients. The recurrence rate of OC patients after surgery is as high as 70% [7]. The recurrence and treatment failure of OC are closely related to the resistance to chemotherapy drugs. Therefore, finding new therapies for OC treatment is significant to reduce the death rate and prolong the survival time of OC patients.

The article "SPOCK2 Promotes the Malignant Behavior of Ovarian Cancer via Regulation of the Wnt/β-Catenin Signaling Pathway" was retracted in 2024. Reasons: signs of a paper mill; suspected computer-generated content; unreliable results or conclusions; concerns about the data.

SPOCK family proteins are proteoglycans of the vertebrate extracellular matrix (ECM) [8]. SPOCK-encoded proteins are capable of participating in a variety of physiological and pathological cellular processes, including tumor progression [9], epithelial-mesenchymal transition [10], and Alzheimer's disease [11], which are hallmarks of both pathological processes such as cancer cell invasion and normal physiological processes such as morphogenesis and differentiation. SPOCK2, also known as Testin-2, is a member of the SPOCK family. Abnormal expression of this gene has been associated with the development of several diseases, and SPOCK2 has been found to be abnormally expressed in lung adenocarcinoma [12], breast [13], and Endometrial cancers [14]. In this study, we examined the role of the SPCOK2 gene in ovarian cancer and preliminarily investigated the relevance of the SPOCK2 gene to the development of ovarian cancer.

## 2. Materials and Methods

### 2.1. Clinical Specimens

54 OC Patients Who Underwent Tumor Resection from January 2015 to January 2017 at Our Hospital Were Selected. All Specimens Taken from the Adjacent Normal Tissues and the Cancer Tissues Were Stored at -80°C for Further Experiments

### 2.2. Cell Lines

OVCAR3, SKOV3, A2780, OV90, and ES-2 were cultured in DMEM medium (Invitrogen, Carlsbad, CA, USA) containing 10% FBS (Invitrogen) and stored in a humidified incubator at 37°C with 5% CO_2_.

### 2.3. Clinical Prognosis Analysis from a Public Database

The online tool GEPIA (http://gepia.cancer-pku.cn/) was used to analyze the SPOCK2 levels between OC tissues and normal tissues. Additionally, OS and DFS analyses of OC patients in the database were downloaded from the website.

### 2.4. Plasmid Construction and Cell Transfection

Cell transfection with si-SPOCK2 or control siRNA was performed with Lipofectamine 2000 (Invitrogen). SPOCK2 overexpression was achieved by transfection of SPOCK2 expression plasmids.

### 2.5. qRT-PCR

Total RNA was isolated with Trizol reagent (Invitrogen), and cDNA was synthesized with a reverse transcription Kit (TaKaRa, Dalian, China). The qRT-PCR assay was performed using SYBR Green (Takara) on an ABI 7500 system. GAPDH was an internal control.

The article "SPOCK2 Promotes the Malignant Behavior of Ovarian Cancer via Regulation of the Wnt/β-Catenin Signaling Pathway" was retracted in 2024. Reasons: signs of a paper mill; suspected computer-generated content; unreliable results or conclusions; concerns about the data.

### 2.6. CCK-8 Assay

Cells transfected with corresponding vectors were cultured at densities of 2 × 103 cells/well. CCK-8 was added into the wells at the indicated time (24, 48, 72, and 96 h) and incubated for 2 h. The OD_450_ was estimated using a microplate reader.

### 2.7. Western Blotting

After measuring protein concentrations using a BCA assay (Beyotime Biotechnology, Jiangsu, China), the samples were separated on SDS-PAGE gels and transferred onto PVDF membranes (Millipore, Billerica, USA). The membranes were blocked with 5% skim milk and then incubated with primary antibodies at 4°C overnight. The antibodies included antibodies for SPOCK2, cleaved caspase-3, procaspase-3, *β*-catenin, c-Myc, cyclin D1, E-cadherin, N-cadherin, Vimentin, and GAPDH (1 : 1000, Abcam). Following 3 washes with TBST, the membranes were incubated with HRP-conjugated secondary antibodies for 1 h at room temperature. GAPDH was an internal control.

### 2.8. Cell Apoptosis Assay

Cell apoptosis was detected by Annexin V-FITC kit (BD Biosciences, USA). The cells were incubated with Annexin V-FITC and PI at room temperature and protected from light for 30 minutes.

### 2.9. Transwell Assay

For cell invasion assays, cells in serum-free DMEM were added into the upper chamber with matrigel on the filter membrane. After incubation for 24 h in 5% CO_2_ at 37°C, the cells that had adhered to the lower membrane were fixed and stained with 20% methanol and 0.1% crystal violet. The cells were counted under an inverted light microscope (Olympus Corporation, Tokyo, Japan). For migration assay, the transwell chamber was not coated with matrigel.

### 2.10. Statistical Analysis

The data were analyzed using SPSS 18.0. The difference was analyzed by Student's *t*-test or by one-way analysis of variance (ANOVA) between two groups or in more than two groups. *χ*^2^ analysis was used to analyze the correlation between JARID2 expressions and clinicopathologic features. *P* < 0.05 was considered statistically significant.

## 3. Results

### 3.1. Expression of SPOCK2 Was Upregulated in Human OC

To confirm the functions of SPOCK2 in OC progression, we examined the expressions of SPOCK2 in OC tissues and cells. The comparison of the expressions of SPOCK2 in OC and normal tissues based on the GEPIA database indicated that SPOCK2 expressions were increased in OC tumors (Figure 1(a)). Similarly, the results of this study also demonstrated the upregulated expressions of SPOCK2 in OC tissues (Figure 1(b)). To further confirm the results, the SPOCK2 expressions in OC cells were examined. Similarly, significantly high SPOCK2 expressions were also identified in OC cells (Figures 1(c) and 1(d)).

The article "SPOCK2 Promotes the Malignant Behavior of Ovarian Cancer via Regulation of the Wnt/β-Catenin Signaling Pathway" was retracted in 2024. Reasons: signs of a paper mill; suspected computer-generated content; unreliable results or conclusions; concerns about the data.

### 3.2. SPOCK2 Overexpression Predicted a Poor Prognosis of OC

To further evaluate the clinical significance of SPOCK2 in OC, we analyzed the relationship between SPOCK2 expressions and clinicopathological characteristics of OC patients. We found significant correlations between SPOCK2 overexpression and TNM stage, lymphoid metastasis, distant metastasis, and FIGO stage (Table 1). No evident correlation was observed between SPOCK2 levels and other clinicopathological features. Furthermore, the prognosis analysis of SPOCK2 in OC patients from the TCGA database also showed that the survival rate of OC patients was markedly decreased in patients with high SPOCK2 expression (Figure 2).

### 3.3. Knockdown of SPOCK2 Suppressed OC Cell Viability

To further determine the functions of SPOCK2 in OC progression, SPOCK2 was silenced by si-SPOCK2 in OC cells. The successful knockdown of SPOCK2 in OC cells was confirmed by RT-qPCR and western blot (Figures 3(a) and 3(b)). CCK-8 assay was used to verify the effect of SPOCK2 in OC cells. The results indicated that the proliferation of OVCAR3 and SKOV3 cells was significantly restrained after SPOCK2 knockdown (Figures 3(c) and 3(d)).

### 3.4. SPOCK2 Downregulation Increased OC Cell Apoptosis

Apoptosis plays a key role in tumor regression, and cell apoptosis was assessed to confirm whether SPOCK2 was involved in OC cell apoptosis. Results of flow cytometric analysis demonstrated that SPOCK2 silence significantly increased the apoptosis rates of OC cells (Figures 4(a) and 4(b)). Furthermore, to elucidate the apoptotic mechanisms of SPOCK2 in OC cells, we detected the levels of caspase-3. Significant upregulation of cleaved caspase-3 was observed in SPOCK2-silenced OC cells, but there were no notable changes in total caspase-3 (Figure 4(c)). These results showed that SPOCK2 downregulation induced OC cell apoptosis through regulation of apoptosis-related proteins.

### 3.5. Downregulation of SPOCK2 Restrained OC Cell Migration and Invasion

To verify the functions of SPOCK2 in OC cells, we performed transwell assays to determine whether SPOCK2 could affect OC cell migration and invasion. As shown in Figure 5(a), migration and invasion of OVCAR3 cells were significantly suppressed, when SPOCK2 was silenced. Similar results were found in SKOV3 cells with SPOCK2 silence (Figure 5(b)). All the above data suggested that SPOCK2 promoted the invasion and metastasis of OC cells.

### 3.6. Upregulation of SPOCK2 Promoted OC Cell Proliferation, Invasion, and Migration

To further confirm the functions of SPOCK2 in OC progression, the SPOCK2 was upregulated in A2780 cells. As shown in Figure 6(a), the successful overexpression of SPOCK2 in A2780 cells was confirmed by RT-qPCR. Then, the proliferation of A2780 cells was examined by CCK-8 assays. Results showed that SPOCK2 upregulation significantly accelerated the proliferation of A2780 cells (Figure 6(b)). Similarly, the functions of SPOCK2 upregulation in A2780 invasion and migration were also detected by transwell assays. We found that A2780 cell invasion and migration were markedly promoted by SPOCK2 overexpression (Figures 6(c) and 6(d)).

The article "SPOCK2 Promotes the Malignant Behavior of Ovarian Cancer via Regulation of the Wnt/β-Catenin Signaling Pathway" was retracted in 2024. Reasons: signs of a paper mill; suspected computer-generated content; unreliable results or conclusions; concerns about the data.

### 3.7. SPOCK2 Promoted OC via Wnt/*β*-Catenin Signaling

To elucidate the potential mechanism of SPOCK2 in OC progression, we analyzed whether the Wnt/*β*-catenin pathway was crucial for OC development. The expressions of activated *β*-catenin, cyclin D1, and c-Myc in OVCAR3 cells were determined, when SPOCK2 was silenced or overexpressed. As shown in Figure 7(a), activated *β*-catenin, cyclin D1, and c-Myc were significantly upregulated by SPOCK2 overexpression and decreased by SPOCK2 knockdown. Furthermore, we also detected the changes in the biological behaviors of OVCAR3 cells transfected with the SPOCK2 vector in the absence or presence of XAV-939, a specific inhibitor of Wnt/*β*-catenin signaling. Results showed that SPOCK2 overexpression remarkably promoted OC cell proliferation, invasion, and migration; the above effects of SPOCK2 were partially eliminated by XAV-939 (Figures 7(b)to 7(d)). These findings indicated that SPOCK2 activated the Wnt/*β*-catenin pathway, finally regulating OC progression.

## 4. Discussion

The incidence of ovarian malignancies has gradually increased in recent years, ranking third among gynecologic tumors, but its mortality rate ranks first among gynecologic tumors [15]. Unless significant progress has been made in ovarian cancer, the prognosis remains poor [16]. Therefore, it is significant to explore new therapies for OC to improve survival. Targeted therapy is a new therapy developed in recent years for the treatment of malignant tumors, which refers to the design of corresponding drugs against well-defined oncogenic protein molecules or gene fragments [17]. Targeted therapy causes specific death of cancer cells by binding targeted drugs to specific cancer sites without affecting surrounding normal tissue cells [18]. Currently, targeted therapeutic agents that have been used in ovarian cancer include olaparib and niraparib, VEGF inhibitors, and the antiangiogenesis inhibitor bevacizumab, but the above-targeted agents are less used in clinical practice because of their narrow indications, high prices, and certain adverse effects [19–21]. Exploring the molecular mechanisms associated with ovarian cancer progression is the basis for developing novel diagnostic and therapeutic approaches for ovarian cancer.

The article "SPOCK2 Promotes the Malignant Behavior of Ovarian Cancer via Regulation of the Wnt/β-Catenin Signaling Pathway" was retracted in 2024. Reasons: signs of a paper mill; suspected computer-generated content; unreliable results or conclusions; concerns about the data.

Previous studies showed that SPOCK presented high plasma levels in multiple cancers and could promote tumor growth, metastasis, and invasion through PI3K/Akt, Wnt/*β*-catenin, and other pathways, and increase cancer cell resistance to chemotherapeutic drugs [22, 23]. In contrast, the role of SPOCK2 in tumors has been less studied. The oligonucleotide polymorphisms of the SPOCK2 gene were associated with chromosome 16q deletion in breast cancer [24]. Sambuudash et al. found that the prevalence of SPOCK2 methylation was markedly increased in colon carcinoma than in normal mucosal tissues, suggesting that methylation of this gene may be associated with colon cancer development [25]. In addition, another study has shown that SPOCK2 plays a crucial role in prostate cancer development by inhibiting the invasion and metastasis of prostate cancer cells [26].

Our previous imaging genomics findings suggested that SPOCK2 was aberrantly expressed in OC. In this study, the expressions of SPOCK2 in OC tissues were significantly higher than that of normal controls, suggesting that this gene may be associated with the development of OC. This result was consistent with our imaging genomics findings. Moreover, we also find that the higher the level of SPOCK2 expression, the more malignant the OC was. Furthermore, the prognosis analysis of SPOCK2 in OC patients from the TCGA database also showed that the survival rate of OC patients markedly declined in patients with high SPOCK2 expressions. To further explore the roles and mechanism of SPOCK2 in OC progression, we knocked down SPOCK2 in OC cells and examined the proliferation, migration, and invasion abilities. Results indicated that downregulation of SPOCK2 could promote cell apoptosis, and inhibit cell proliferation, migration and invasion. Moreover, activated *β*-catenin, cyclin D1, and c-Myc proteins were reduced after knockdown of SPOCK2, which suggested that SPOCK2 could affect the EMT of OC through Wnt/*β*-catenin, and thus affect the invasion and metastasis of OC. However, the mechanistic studies in the current study are insufficient, such as the functions of SPOCK2 *in vivo*, and whether SPOCK2 exerted functions in OC through regulation of certain downstream molecules, which deserves further exploration.

In conclusion, upregulated SPOCK2 in OC tissues was identified, which was related to poor OC prognosis. Silencing SPOCK2 may inhibit OC cell progression by inactivating Wnt/*β*-catenin, which may provide a reference for the clinical diagnosis and treatment of OC.

The article "SPOCK2 Promotes the Malignant Behavior of Ovarian Cancer via Regulation of the Wnt/β-Catenin Signaling Pathway" was retracted in 2024. Reasons: signs of a paper mill; suspected computer-generated content; unreliable results or conclusions; concerns about the data.

## Figures and Tables

**Figure 1:** SPOCK2 was upregulated in OC tissues and cells. (a) The expression patterns of SPOCK2 in OC tumors and normal OC tissues from the GEPIA database. (b) The mRNA expressions of SPOCK2 in OC tissues and adjacent normal tissues. (c and d) The mRNA and protein expressions of SPOCK2 in OC cells.

**Figure 2:** SPOCK2 overexpression indicated a shorter survival rate for OC patients.

**Figure 3:** Knockdown of SPOCK2 suppressed OC cell viability. (a and b) SPOCK2 was silenced in OC cells. (C, D) SPOCK2 downregulation suppressed OC cell viability.

**Figure 4:** SPOCK2 downregulation increased OC cell apoptosis. (a and b) SPOCK2 silence significantly increased the apoptosis rates of OVCAR3 and SKOV3 cells. (c) Significant upregulation of cleaved caspase-3 was observed in SPOCK2 silenced OC cells.

**Figure 5:** Downregulation of SPOCK2 restrained OC cell migration and invasion. (a and b) OVCAR3 and SKOV3 cell migration and invasion were significantly suppressed, when SPOCK2 was silenced.

**Figure 6:** Upregulation of SPOCK2 promoted OC cell proliferation, invasion, and migration. (a) SPOCK2 was overexpressed in A2780 cells. (b–d) SPOCK2 overexpression promoted A2780 cell proliferation, invasion, and migration.

**Figure 7:** SPOCK2 promoted OC via the Wnt/*β*-catenin signaling pathway. (a) Expression of Wnt/*β*-catenin signaling-related proteins in SPOCK2-overexpressed or -silenced OC cells. (b–d) Wnt/*β*-catenin signaling was involved in the functions of SPOCK2 in OC proliferation, migration, and invasion.

**Table 1:** Correlation of SPOCK2 expression with the clinicopathological characteristics of ovarian cancer patients.

Clinicopathological features	Cases (*n* = 54)	SPOCK2^a^ expression		*P* value
		High (*n* = 27)	Low (*n* = 27)	
Age (years)				0.785
>60	29	14	15	
≤60	25	13	12	
Family history of cancer				0.102
Yes	26	10	16	
No	28	17	11	
Tumor size (cm)				0.112
≥5.0	26	12	17	
<5.0	28	15	10	
TNM stage				0.003^∗^
I-II	29	9	20	
III	25	18	7	
Lymph-node metastasis				0.014^∗^
Yes	25	17	8	
No	29	10	19	
Pausimenia				0.413
Yes	25	11	14	
No	29	16	13	
FIGO stage				0.013^∗^
I-II	31	11	20	
III-IV	23	16	7	
Distant metastasis				0.029^∗^
Yes	28	18	10	
No	26	9	17	

## Data Availability

The datasets used during the current study are available from the corresponding author on reasonable request.
